RETRACTED

# SETDB1 promotes glioblastoma growth via CSF-1-dependent macrophage recruitment by activating the AKT/mTOR signaling pathway

**DOI:** 10.1186/s13046-020-01730-8

**Published:** 2020-10-15

**Authors:** Shuai Han, Wei Zhen, Tongqi Guo, Jianjun Zou, Fuyong Li

**Affiliations:** 1 Department of Neurosurgery, the First Hospital of China Medical University, Shenyang, Liaoning Province China; 2 Department of Neurosurgery, The People’s Hospital of China Medical University (The People’s Hospital of Liaoning Province), No.33, Wenyi Road, Shenhe District, Shenyang, 110016 Liaoning Province PR China

**Keywords:** SETDB1, Glioblastoma, AKT/mTOR, TAMs, CSF-1

## Abstract

**Background:**

Glioblastoma is a common disease of the central nervous system (CNS), with high morbidity and mortality. In the infiltrate in the tumor microenvironment, tumor-associated macrophages (TAMs) are abundant, which are important factors in glioblastoma progression. However, the exact details of TAMs in glioblastoma progression have yet to be determined.

**Methods:**

The clinical relevance of SET domain bifurcated 1 (SETDB1) was analyzed by immunohistochemistry, real-time PCR and Western blotting of glioblastoma tissues. SETDB1-induced cell proliferation, migration and invasion were investigated by CCK-8 assay, colony formation assay, wound healing and Transwell assay. The relationship between SETDB1 and colony stimulating factor 1 **(**CSF-1), as well as TAMs recruitment was examined by Western blotting, real-time PCR and syngeneic mouse model.

**Results:**

Our findings showed that SETDB1 upregulated in glioblastoma and relative to poor progression. Gain and loss of function approaches showed the SETDB1 overexpression promotes cell proliferation, migration and invasion in glioblastoma cells. However, knockdown SETDB1 exerted opposite effects in vitro. Moreover, SETDB1 promotes AKT/mTOR-dependent CSF-1 induction and secretion, which leads to macrophage recruitment in the tumor, resulted in tumor growth.

**Conclusion:**

Our research clarified that SETDB1 regulates of tumor microenvironment and hence presents a potential therapeutic target for treating glioblastoma.

## Introduction

Glioma is a tumor type that derived from glial cells, with a high incidence, high recurrence rate, and poor prognosis [1]. Previous research has demonstrated that gliomas account for 47.1% of primary malignant brain and other central nervous system tumors, of which glioblastoma is the main type of gliomas, accounting for about 56.1% of cases [2, 3]. The treatment process for glioma includes surgery followed by radiotherapy, with or without temozolomide (TMZ) chemotherapy [4, 5].

Previous studies have shown that the interaction between glioblastoma cells and tumor microenvironment plays an important role in glioblastoma progression [6]. Revealing the underlining mechanism of interaction between glioblastoma cells and tumor microenvironment components may be useful for the discovery of novel therapeutic targets [7, 8]. The tumor microenvironment is comprised of diverse nonmalignant stromal cell types that are associated with tumor progression and metastasis, such as tumor-associated macrophages (TAMs) of the hematopoietic lineage, which are abundant migratory cells [9, 10]. Macrophages roughly develop into two main groups with different functions in immune defense and immune surveillance called classically activated macrophages (M1) and alternatively activated macrophages (M2), both of which can transform into each other with the changes in the internal environment [10, 11]. The density of these cells has been shown to be related to the prognosis of several types of cancer, such as glioblastoma [12, 13]. The heterogeneous nature of these cells and their ability to show different responses to cues from the environment is indicative of their roles in cancer progression [14, 15].

RETRACTED

The microenvironment is modulated by the chemokine profile at the tumor site, as this influences macrophage differentiation to hence affect the advancement of glioblastoma [16, 17]. Among these chemokines, colony stimulating factor 1 (CSF-1) is a ubiquitously produced factor seen in many tumors (including glioblastoma) that is vital for metastasis [18]. This factor causes the recruitment of TAMs and other cell subsets to influence the processes of inflammation, angiogenesis, proliferation and evasion of the immune response [19, 20]. The use of anti-CSF-1 antibodies has been shown to decrease the in vivo tumor burden by 96%, according to preclinical cancer models [21].

SETDB1 (SET domain bifurcated 1) is encoded by the approximately 38.6 kb long *SETDB1* gene located on human chromosome 1q21.3 [22]. This protein is a member of the methyltransferase family of SET-domains (Su (var)3–9, E(z), Trithorax) that function by silencing genes or inhibiting transcription via H3K9 trimethylation [23]. SETDB1 is linked to embryonic development and is also a candidate for early Huntington disease therapy. Recently, research pointed out that SETDB1 is expressed at abnormal and high levels in melanoma, ovarian cancer, lung cancer, and breast cancer [24–28]. The involvement and function of SETDB1 in glioblastoma have yet to be well studied, which calls for studies in this direction.

In the current study, we identified that SETDB1 was markedly upregulated in glioblastoma and displayed a significant association with the clinicopathological characteristics and survival of glioblastoma patients. Overexpressing SETDB1 boosted the transcription of CSF-1 by activating the AKT/mTOR signaling pathway. Furthermore, SETDB1 induced CSF-1 expression in glioblastoma cells leading to the recruitment of TAMs and subsequent tumor growth. These finding indicate the role of SETDB1 in both oncogenesis and TAM recruitment in glioblastoma pathogenesis.

RETRACTED

## Material and methods

### Cell culture and reagents

American Type Culture Collection (ATCC, Manassas, VA, USA) was the source of glioblastoma cell lines: U87, U251, H4, A172, U118, LN229, SHG-44 and GL261. Cell culture was performed in Dulbecco’s modified Eagle’s medium (DMEM) with 10% fetal bovine serum (FBS), 100 U/mL penicillin and 100 μg/mL streptomycin (HyClone, Thermo, USA) at 37 °C and 5% CO_2_. NHAs (Normal human astrocytes) were procured from Lonza (Switzerland) and cultured as per supplied instructions. Rapamycin (Selleckchem) and MK-2206 (Selleckchem) were diluted with DMSO (Sigma).

### Human glioblastoma samples

Glioblastoma tissues (*n* = 40) and neighboring healthy tissues (n = 40) were surgically excised at The People’s Hospital of China Medical University and the First Hospital of China Medical University. Table 1 displays the clinicopathological features of the patients. Regular follow-up was performed for patients along with informed consent. Other data included relapse-free survival and overall survival (OS). This work received approval from the ethics committee of The People’s Hospital of China Medical University and the First Hospital of China Medical University.

**Table 1:** Clinicopathologic Features of SETDB1 expression in glioblastoma

	Low SETDB1 level (*n* = 40)	High SETDB1 level (n = 40)	*p* value
**Age**	55 ± 13.33	57 ± 12.65	0.432
**Gender**			0.469
Male	24	29	
Female	16	11	
**TNM stage**			0.001
I, II	32	7	
III, IV	8	33	

### Immunohistochemistry (IHC)

In accordance with previous works [29, 30], staining of tissues was performed with a SETDB1 antibody (Sigma-Aldrich, USA). The scoring of cells was performed in accordance with the following guide: 0 (no positive staining); 1 (1 to 25% positive cells); 2 (26 to 50% positive cells); 3 (51 to 75% positive cells); and 4 (> 75% positive cells). The scoring for staining intensity was performed as follows: 0, negative; 1, weak; 2, moderate; and 3, high. The formula for SETDB1-positive cells was as follows: staining intensity score × percentage. This score involved both the nucleus and cytoplasm and was analyzed by two pathologists.

### Cell invasion assay

The migration assay used Falcon cell culture inserts from BD (Franklin, USA). The invasion assay utilized a BioCoat™ Matrigel™ Invasion Chamber (BD) in accordance with the instructions of the manufacturer. A phase contrast microscope was utilized to count cells; the average of 5 various fields/well was considered.

RETRACTED

### Wound-healing assay

Indicated ells were cultured in 6-well plates in triplicate for each cell line until approximately 90% confluent. Wounds were made in each confluent monolayer of cells with a sterile 200-μl pipette tip, and fresh growth medium was replaced. Microscopic pictures were taken of the same field at 24 h.

### Macrophage migration assay

The 24-well transwell plates (Corning Inc) were used to examine the macrophages migration induced by CM from U87 cells with indicated treatment. Macrophages were collected and added into the top chamber of 24-well transwell plates. Simultaneously, CM were added into the bottom of transwell chamber. After 24 h, the cells that crossed the inserts were stained with crystal violet and counted under phase-contrast microscopy.

### CCK-8 assay

The indicated cells (5000 per well) were plated in 96-well plates and grown in normal culture conditions. Cell proliferation was determined every 24 h for 4 days using a CCK-8 assay.

### Clone formation assay

Six-well plates were used to plate single-cell suspensions at a density of 1000 cells per plate. Every 3 days, the culture medium was replaced. After allowing 2 weeks for clone formation, fixation and staining of the clones was performed using 0.1% crystal violet/40% methanol. Microscopy was performed to count colonies with > 50 cells/colony.

### RNA extraction and real-time PCR

Real-time PCR was performed as previously described [31, 32]. Briefly, TRIzol (Invitrogen, USA) was utilized for the extraction of total RNA. cDNA was synthesized with the PrimeScript™ RT reagent kit (Takara, Dalian) in accordance with the instructions of the manufacturer. SYBR Premix ExTaq II (Takara, Dalian) was utilized for real-time PCR of this cDNA on an ABI PRISM 7300 (Applied Biosystems, USA) to analyze the chemokines of the immune system. GAPDH was used to normalize mRNA levels. The primers used are listed in Table 2.

**Table 2:** Real-time PCR primers

SETDB1	Forward	5′-GGAGGAACTTCGTCAGTACATTG-3′
	Reverse	5′-TCTTTCTGTAGTACCCACGTCTC-3′
CSF-1	Forward	5′-AGTATTGCCAAGGAGGTGTCAG-3′
	Reverse	5′-ATCTGGCATGAAGTCTCCATTT-3′
TGF-β	Forward	5′-AAGAAGTCACCCGCGTGCTA-3′
	Reverse	5′-TGTGTGATGTCTTTGGTTTTGTCA-3′
IL-8	Forward	5′-GTGCAGTTTTGCCAAGGAGT-3′
	Reverse	5′-TTATGAATTCTCAGCCCTCTTCAAAAACTTCTC-3′
IL-4	Forward	5′-CCGTAACAGACATCTTTGCTGCC-3′
	Reverse	5′-GAGTGTCCTTCTCATGGTGGCT-3′
IL-13	Forward	5′-CCTCTGACCCTTAAGGAGCTTAT-3′
	Reverse	5′-CGTTGCACAGGGGAGTCTT-3′
VEGF	Forward	5′-CAAGCCAAGGCGGTGAGCCA-3′
	Reverse	5′-TCTGCCGGAGTCTCGCCCTC-3′
CCL2	Forward	5′-AGGTGTCCCAAAGAAGCTGTA-3′
	Reverse	5′-ATGTCTGGACCCATTCCTTCT-3′
CCL20	Forward	5′-TCCTGGCTGCTTTGATGTCA-3′
	Reverse	5′-CAAAGTTGCTTGCTGCTTCTGA-3′
CD86	Forward	5′-TCTCCACGGAAACAGCATCT-3′
	Reverse	5′-CTTACGGAAGCACCCATGAT-3′
CD163	Forward	5′-TCCACACGTCCAGAACAGTC-3′
	Reverse	5′-CCTTGGAAACAGAGACAGGC-3′
IL-10	Forward	5′-ATGCTGCCTGCTCTTACTGACTG-3′
	Reverse	5′-CCCAAGTAACCCTTAAAGTCCTGC-3′
CCL17	Forward	5′-AGGGACCTGCACACAGAGAC-3′
	Reverse	5′-AGGTAGTCCCGGGAGACAGT-3′
CCL22	Forward	5′-TGCCATCACGTTTAGTGAAGG-3′
	Reverse	5′-CGGCAGGATTTTGAGGTCCA-3′
GAPDH	Forward	5′-AATGGATTTGGACGCATTGGT-3′
	Reverse	5′-TTTGCACTGGTACGTGTTGAT-3′

RETRACTED

### Transfection and knockdown

Transfections with targeted siRNA against *AKT* were performed using lipofectamine 3000 according to the manufacturer’s instructions. Stable *SETDB1* knockdown cells were generated by transducing U87 or U251 cells with the pLKO.1-puro lentiviral vector (Addgene) expressing shRNA. Lentiviral particles were generated by co-transfecting 293 T cells with the lentiviral vector, pMD2.G (VSVG), pMDLg/pRRE, and pRSV-REV (Addgene). Following lentiviral transduction, cells were plated in 96-well plates in the presence of puromycin (2 μg/ml; EMD/Millipore). SETDB1 expression of the puromycin-resistant clones was then analyzed by Western blotting. The sequences are listed in Table 3.

**Table 3:** Knockdown sequence

	Target sequence
si AKT	GGAGGGUUGGCUGCACAAA
sh SETDB1	GGTGATGAGTACTTTGCCA

### Western blotting

Western blotting was performed as previously described [33, 34]. Briefly, cell lysis was performed with the RIPA buffer protein extraction reagent (Pierce, Rockford, IL, USA) containing a protease inhibitor cocktail (Roche, USA). The proteins were resolved by 10% SDS-PAGE followed by transfer to polyvinylidene fluoride (PVDF) membranes (Sigma-Aldrich). Next, the membranes were blocked using 5% bovine serum albumin (BSA) and incubated with primary antibodies at 4 °C overnight. Appropriate secondary antibodies were later added and then visualized by using an ECL chemiluminescence kit. The primary antibodies used are listed as follows: SETDB1 (HPA018142, Sigma-Aldrich), cleaved caspase 3 (9661, Cell signaling technology), cleaved caspase 8 (9748, Cell signaling technology), slug (9585, Cell signaling technology), vimentin (5741, Cell signaling technology), E-cadherin (14,472, Cell signaling technology), mTOR (2983, Cell signaling technology), p-mTOR (5536, Cell signaling technology), AKT (4685, Cell signaling technology), p-AKT (4060, Cell signaling technology), CSF-1 (3155, Cell signaling technology), β-actin (3700, Cell signaling technology).

RETRACTED

### Macrophage cells isolation and differentiation

The preparation of human monocytes from buffy coats of healthy volunteers was performed using Ficoll-Hypaque (Pharmacia Corporation) for 50 min at 400 g. Twenty-four-well plates were seeded with 2 × 10^6^ cells/mL in RPMI 1640 medium containing 10% heat inactivated human AB serum, 50 U of penicillin/mL, 50 U of streptomycin/mL, 2 mM L-glutamine, and 100 ng/mL human M-CSF (which allows differentiation into macrophages). Warm medium was used to gently wash away non-adherent cells 6 days post-culture. CD14^+^ macrophages were found to account for greater than 95% of the adherent cells. The activation of these monocytes to macrophages in vitro involved the treatment of 2 × 10^6^ cells/L with 25 μg/mL lipopolysaccharide (LPS, Sigma-Aldrich) to produce M1-polarized macrophages and 45 ng/mL recombinant human interleukin-4 (IL-4; R&D) to produce M2-polarized macrophages. Flow cytometry was employed to detect the formation of macrophages. For the following in vitro assays, cells were cultured for 24 h with RPMI media minus supplements and meticulously washed with PBS prior to the experiments.

### Animal experiments

For the xenograft model, 5 × 10^5^ U251-EV, U251-SETDB1, U87-shCon or sh*SETDB1* cells in 100 μL of PBS was performed followed by subcutaneous injection in the flanks of nude mice. The mice were sacrificed 15 days and tumor weights were assessed. The mice were kept at the Mouse Experimentation Core premises of the China Medical University.

The syngeneic glioblastoma mouse model was generated in accordance with previous reports [35, 36]. Briefly, 2% isoflurane in O_2_ was used to sedate C57BL/6 J mice (4–6 weeks old). The addition of 5 × 10^5^ GL261-EV and GL261-SETDB1 cells in 100 μL of PBS was performed followed by subcutaneous injection in the flanks of C57BL/6 J mice. The mice were sacrificed after 19 days and tumor weights were assessed.

### Statistical analysis

The mean ± standard deviation (SD) was used to represent the data of triplicate assays. Student’s *t-*test was applied to assess significant differences between groups. Repeated measures analysis of variance was performed to assess variations between tumor parameters (growth rate and cell growth) of the animals.

## Results

### SETDB1 is frequently overexpressed and predicts poor glioblastoma prognosis

To investigate the role of SETDB1 in glioblastoma cells, the level of SETDB1 was assessed in glioblastoma patients. IHC and real-time PCR results demonstrated that SETDB1 was evidently increased in tumor samples compared with surrounding healthy tissues (Fig. 1a and b). Next, western blotting was employed to assess the protein level of SETDB1 in cell lines. Higher levels of SETDB1 were detected in the glioblastoma cells in comparison with NHAs (Fig. 1c). In addition, real-time PCR result showed that SETDB1 mRNA level was higher in glioblastoma cells than in NHAs cells (Fig. 1d).

RETRACTED

**Fig. 1:** SETDB1 was upregulated in glioblastoma tissues and corelative with poor tumor progression. **a** Representative IHC staining of SETDB1 protein expression in glioblastoma tumor tissues (T) and adjacent normal tissue (N) of three patients. Scale bar: 50 μm. **b** mRNA level of SETDB1 was analyzed by real-time PCR in glioblastoma tumor tissues (T) and adjacent normal tissue (N) of patients. **c** Western blotting of SETDB1 expression in NHAs and indicated glioblastoma cells. **d** mRNA level of SETDB1 was analyzed by real-time PCR in NHAs and indicated glioblastoma cells. **e** Kaplan-Meier survival analysis indicated that glioblastoma patients with high expression of SETDB1 had worse relapse-free survival

This was followed by studying the effect of this SETDB1 overexpression in the clinic. Increased mRNA expression of SETDB1 was evidently linked to shorter relapse-free glioblastoma survival, as shown by Kaplan-Meier curves (*p* = 0.025; Fig. 1e). Our findings indicate that age and sex had no association with SETDB1 expression and TNM stage were found to be linked with the protein expression (Table 1). SETDB1 was also found to serve as an independent factor for prognosis and shorter relapse-free survival, as shown by the multivariate Cox regression analysis (Table 4). Overall, high expression of SETDB1 was found to serve as a prognostic factor for glioblastoma.

**Table 4:** Cox regression analysis for relapse-free survival in glioblastoma patients

	Univariate analysis		Multivariate analysis	
	Hazard ratio (95% CI)	*p* value	Hazard ratio (95% CI)	*p* value
SETDB1 expression (high vs. low)	2.234 (0.981–4.128)	0.023	2.459 (1.232–5.483)	0.018
Age	1.321 (0.548–2.325)	0.563	1.431 (0.674–2.543)	0.554
Male vs. Female	1.453 (0.674–3.092)	0.345	1.543 (0.783–3.482)	0.323
Stage (III, IV vs. I. II)	1.982 (1.128–3.763)	0.007	1.889 (1.093–3.542)	0.011

### SETDB1 enhances the growth of glioblastoma and inhibits apoptosis

We next investigated the biological functions of SETDB1 involved in U87 and U251 cells. We overexpression or knockdown SETDB1 in U87 and U251 cells with lenti-SETDB1, Lentiviruses with empty vector (EV), sh SETDB1 or negative control shRNA (shCon) transfection. The following changes in expression were assessed using real-time PCR and Western blotting (Fig. 2a, b, S1A and S1B). Increased SETDB1 expression caused an evident increase in proliferation and clone formation in the cell lines studied compared with those in the controls (Fig. 2c and d). SETDB1 silencing caused the opposite results: decreased cell division and clone formation (Fig. S1C-S1F). Next, the effect of this ectopic expression on apoptosis was studies; increased expression of SETDB1 noticeably reduced the levels of the active (cleaved) forms of caspase-8 and caspase-3 and hence decreased apoptosis in the cell lines mentioned previously in the presence or absence of staurosporine (STS) or TRAIL (Fig. 2e and S1G). The opposite results were seen when silencing SETDB1, as indicated by increased sensitivity to STS or TRAIL treatment and increased apoptosis and expression of its markers in U251 cells (Fig. S1H and S1I).

RETRACTED

**Fig. 2:** SETDB1 promotes cell growth, and apoptosis in vitro and in vivo. **a** mRNA level of SETDB1 in indicated cells transfected with SETDB1 plasmid or control vector. **b** Western blotting of SETDB1 in indicated cells transfected with SETDB1 plasmid or control vector. **c** CCK-8 of indicated cells transfected with SETDB1 plasmid or control vector. **d** Colony formation of indicated cells transfected with SETDB1 plasmid or control vector. **e** Western blotting of indicated proteins in U251 cells transfected with SETDB1 plasmid or control vector treated with 500 nM staurosporine (STS) for 24 h. **f** Ectopic expression of SETDB1 accelerated growth of U251 xenografts in nude mice (*n* = 6) as compared to controls. **g** Western blotting of ectopic expression of SETDB1 in tumors from U251-SETDB1 groups. **h** Representative images of Ki67-positive cells in vector and SETDB1 transfected tumors. Scale bar: 50 μm. Results were expressed as means ± SD of 3 independent experiments. **, *P* < 0.01

Further investigation involved the subcutaneous injection of U251-EV and U251-SETDB1 into nude mice. This ectopic SETDB1 expression caused a conspicuous growth increase in tumors in the animals (Fig. 2f). SETDB1 overexpression was confirmed by Western blotting (Fig. 2g). Ki-67 assays showed that U251-SETDB1 xenografts displayed increased numbers of proliferating cells (Fig. 2h). However, knockdown of SETDB1 caused an evident decrease in xenograft size (Fig. S1J and S1K). Markedly decreased cell proliferation was observed in U87-sh*SETDB1* xenografts according to Ki-67 staining results (Fig. S1L). Overall, SETDB1 is vital in the oncogenesis and advancement of glioblastoma.

### SETDB1 increases migration and invasion in glioblastoma cells

Assays to assess the abilities of cells to migrate and invade were performed to examine the metastasis potential in vitro. The ability of cells to migrate and invade was augmented in the presence of ectopic SETDB1 expression in the U87 and U251 cell lines compared with the control (Fig. 3a and b). Upregulation of Slug and Vimentin (mesenchymal markers) and downregulation of E-cadherin (an epithelial marker) were shown by western blotting (Fig. 3c). The opposite results were observed for the same cell lines that were subjected to silencing of SETDB1, which decreased the ability of the cells to invade (Fig. 3d and e), decreased Slug and Vimentin and increased E-cadherin (Fig. 3f). Moreover, overexpression of SETDB1 in stable SETDB1 cells attenuated SETDB1 silencing-induced invasion, migration suppression and EMT regulation (Fig. 3d-f). The above data suggest that SETDB1 regulates migration, invasion and EMT in glioblastoma.

RETRACTED

**Fig. 3:** SETDB1 promotes invasion, migration and EMT of glioblastoma cells. **a** Representative images of matrigel invasion assay revealed that ectopic expression of SETDB1 promoted glioblastoma cells invasion. Scale bar: 100 μm. **b** Representative images of wound-healing assay indicated that ectopic expression of SETDB1 promoted cell migration in glioblastoma cells. Scale bar: 100 μm. **c** Western blotting of mesenchymal markers (Slug and Vimentin) and epithelial markers (E-cadherin) in cells transfected with SETDB1 or control plasmid. Scale bar: 100 μm. **d** Representative images of matrigel invasion assay revealed that downregulation of SETDB1 suppressed glioblastoma cells invasion. Scale bar: 100 μm. **e** Representative images of wound-healing assay indicated that downregulation of SETDB1 suppressed cell migration in glioblastoma cells. **f** Western blotting of mesenchymal markers (Slug and Vimentin) and epithelial markers (E-cadherin) in cells transfected with stable shRNA against *SETDB1*. Results were expressed as means ± SD of 3 independent experiments. **, *P* < 0.01

### Increased SETDB1 promotes CSF-1 secretion from glioblastoma

The levels of cytokines and chemokines CSF-1, TGF-β, IL-4, IL-13, and VEGF involved in the infiltration of TAMs were assessed through real-time PCR for SETDB1 in glioblastoma lines. U87 and U251 glioblastoma cells displayed elevated profiles of CSF-1 mRNA and proteins in the presence of SETDB1 overexpression (Fig. 4a and b**)**, while knockdown caused the opposite effects (Fig. 4c and d). In addition, the ELISA demonstrated that SETDB1 promotes CSF-1 secretion (Fig. 4e), as well as SETDB1 knockdown suppresses CSF-1 secretion (Fig. 4f). As expected, CSF-1 expression significantly correlated with CD163 and SETDB1 expression in glioblastoma samples (Fig. 4g and h). These observations are indicative of higher CSF-1 secretion due to elevated levels of SETDB1, which is in turn connected to increased TAMs in glioblastoma.

RETRACTED

**Fig. 4:** SETDB1 regulates CSF-1 level in glioblastoma cells. **a** Real-time PCR for mRNA level of genes coding for tumor-associated macrophage (TAMs) recruitment associated cytokines in U87 cells with SETDB1 overexpression. **b** Real-time PCR for mRNA level of genes coding for tumor-associated macrophage (TAMs) recruitment associated cytokines in U251 cells with SETDB1 overexpression. **c** Real-time PCR for mRNA level of genes coding for tumor-associated macrophage (TAMs) recruitment associated cytokines in U87 cells with SETDB1 knockdown. **d** Real-time PCR for mRNA level of genes coding for tumor-associated macrophage (TAMs) recruitment associated cytokines in U251 cells with SETDB1 knockdown. **e** Enzyme-linked immunosorbent assay (ELISA) analysis of CSF-1 concentration in the supernatants of cultured glioblastoma cells with SETDB1 overexpression. **f** Enzyme-linked immunosorbent assay (ELISA) analysis of CSF-1 concentration in the supernatants of cultured glioblastoma cells with SETDB1 knockdown. **g** TCGA database indicated the correlation of CD163 and CSF-1 in glioblastoma tissues. **h** TCGA database indicated the correlation of SETDB1 and CSF-1 in glioblastoma tissues. Results were expressed as means ± SD of 3 independent experiments. **, *P* < 0.01

### SETDB1 promoted the secretion of CSF-1 by activating the AKT/mTOR signaling pathway

Next, the potential involvement of the AKT/mTOR signaling pathway in the CSF-1 secretion caused by SETDB1 was assessed. Increased AKT and mTOR phosphorylation was shown by Western blotting when SETDB1 was overexpressed in glioblastoma lines, and this effect was reversed by administration of MK-2206 (Fig. 5a and b). Similarly, knockdown of AKT expression using siRNA attenuated the increase of CSF-1 due to SETDB1 overexpression (Fig. 5c and d). Moreover, Rapamycin, a mTOR inhibitor, attenuated SETDB1-induced CSF-1 upregulation in U87 and U251 cells (Fig. 5e and f). To decipher the SETDB1/AKT/mTOR/CSF-1 axis in vivo, we performed Western blotting analysis on the tumor tissue from the xenograft model. We found that SETDB1 knockdown significantly reduced AKT activation and CSF-1 protein expression in the xenograft model, while SETDB1 overexpression remarkably promoted AKT activation and CSF-1 protein levels in xenograft tumor tissues (Fig. 5g and h). Overall, these observations suggest the involvement of AKT/mTOR signaling in the increase in SETDB1-mediated CSF-1 synthesis. Hence, this axis can serve as a prognostic marker in patients.

**Fig. 5:** PI3K/AKT signaling pathway mediated SETDB1-induced CSF-1 induction. **a** Western blotting of indicated proteins in U87 cells transfected with SETDB1 overexpression with or without MK-2206 pretreatment. **b** Western blotting of indicated proteins in U251 cells transfected with SETDB1 overexpression with or without MK-2206 pretreatment. **c** Western blotting of indicated proteins in U87 cells transfected with SETDB1 overexpression with or without siRNA against *AKT*. **d** Western blotting of indicated proteins in U251 cells transfected with SETDB1 overexpression with or without siRNA against *AKT*. **e** Western blotting of indicated proteins in U87 cells transfected with SETDB1 overexpression with or without rapamycin pretreatment. **f** Western blotting of indicated proteins in U251 cells transfected with SETDB1 overexpression with or without rapamycin pretreatment. **g** Western blotting of indicated proteins in control and SETDB1 overexpression xenograft tumors. **h** Western blotting of indicated proteins in control and SETDB1 knockdown xenograft tumors

RETRACTED

### SETDB1 promotes recruitment and polarization of macrophages via CSF-1

The involvement of this SETDB1-CSF-1 axis in macrophage infiltration was assessed by an in vitro migration assay using conditioned media (CM) from glioblastoma cells overexpressing SETDB1. Compared with control CM, CM from these cells was found to clearly augment the recruitment of macrophages (Fig. 6a). Further, this recruitment was evidently suppressed when a CSF-1 antagonist was administered to macrophages. Overall, these results suggest that macrophage migration is mediated by SETDB1 via CSF-1 induction.

**Fig. 6:** SETDB1 promotes macrophage recruitment and polarization. **a** Transwell migration assay of macrophage by CM from indicated U87 cells. **b** Real-time PCR for the expression levels of CD68 and CD163 in macrophages treated with CM from U87 cells as indicated. **c** Flow cytometry analysis for the expression levels of CD163 in macrophages treated with CM from glioblastoma cells as indicated. **d** Real-time PCR for the mRNA expression of tumor-associated macrophage (TAM) characteristic cytokines in macrophages treated with CM from glioblastoma cells as indicated. **e** Enzyme-linked immunosorbent assay (ELISA) for the secretion of tumor-associated macrophage (TAM) characteristic cytokines in macrophages treated with CM from U87 cells as indicated. **f** Real-time PCR for the mRNA expression of M1-related cytokines in macrophages treated with CM from U87 cells as indicated. **g** Enzyme-linked immunosorbent assay (ELISA) for the secretion of M1-related cytokines in macrophages treated with CM from U87 cells as indicated. Results were expressed as means ± SD of 3 independent experiments. **, *P* < 0.01

Next, the effect of SETDB1 on macrophage polarization via CSF-1 was assessed. The CM from glioblastoma cell lines overexpressing SETDB1 caused elevated expression of CD163 (a M2 macrophage marker) mRNA compared to that in cells cultured with control CM, while there was no change in the expression of CD68 (a M1 macrophage marker) (Fig. 6b). Flow cytometry showed a similar protein profile (Fig. 6c). The cytokine mRNAs and proteins that are representative of TAMs, IL-10, CCL17, and CCL22, were noticeably higher in TAMs incubated with CM from U87 cells with high SETDB1 expression than in TAMs incubated with CM from control cells (Fig. 6d and e). In addition, we also analyzed M1-related genes and found macrophage incubated with CM from SETDB1 overexpression U87 cells does not affect IL-12, IL-23 and CXCL10 levels (Fig. 6f and g). Overall, these data suggest a role for CSF-1 and SETDB1 in promoting macrophage entry and differentiation.

RETRACTED

### SETDB1 promotes tumor growth in a TAM-dependent manner

To demonstrate whether the oncogenic roles of SETDB1 in glioblastoma are TAM-dependent, we investigated the susceptibility of macrophages to liposomal clodronate treatment. For this, we overexpressed SETDB1 in the mouse glioblastoma cell line GL261, which showed faint SETDB1 protein expression (Fig. 7a). Next, we performed a syngeneic mouse model study with injection of SETDB1-overexpressing and control cell lines into the C57BL/6 J mice. Prior to injection, liposomes containing clodronate or PBS were administered for 2 weeks and continued for additional 19 days after tumor implantation (Fig. 7b). The clodronate treatment caused a suppression in mSETDB1-induced F4/80+ macrophages infiltration in the glioblastoma tumors of the animals (Fig. 7c and d). The increased tumor burden induced by SETDB1 overexpression was largely attenuated in mice that received clodronate liposomes (Fig. 7e and f). Moreover, no significant difference in the body weights between these four groups was observed during the course of the experiment (Fig. 7g). The above data suggested that the tumor-promoting effects of SETDB1 in glioblastoma are, at least in part, mediated by macrophage infiltration of the tumor microenvironment.

**Fig. 7:** SETDB1 promotes tumor growth in a macrophage-dependent manner. **a** Western blotting of SETDB1 overexpression efficiency in GL261 cells. **b** Treatment scheme depicting intraperitoneal application of clodronate liposomes or phosphate-buffered saline (PBS) liposomes in C57BL/6 J mice for 4 weeks. GL261 cells were administered at the end of week 2 and animals were sacrificed 2 weeks later. **c** Representative immunohistochemistry of F4/80+ cells in sections from tumors obtained from C57BL/6 J mice treated with clodronate liposomes or PBS liposomes. Scale bar: 50 μm. **d** Tumor volume of vector and SETDB1 overexpression tumors from clodronate-liposome or PBS-liposome-treated mice (*n* = 6 per group). **e** Tumor weight of vector and SETDB1 overexpression tumors from clodronate-liposome or PBS-liposome-treated mice (n = 6 per group). **g** The body weight of mice of indicated groups. **h** A working model of how SETDB1 regulates TAMs recruitment and tumor growth in glioblastoma

RETRACTED

## Discussion

The progression of glioblastoma involves the role of interconnected glioblastoma cells and TAMs in the tumor microenvironment [37]. This increase in infiltrates is connected to the poor prognosis of glioblastoma [5]. The function of this system is yet to be characterized; thus, further studies are warranted to identify such patterns to rapidly unearth potential molecules that may serve as therapeutic tools [13]. In the current study, we revealed that SETDB1 is involved in the modulation of the tumor microenvironment of glioblastoma progression. SETDB1 was found to promote CSF-1 expression and secretion by activating the AKT/mTOR pathway. Moreover, SETDB1-induced CSF-1 modulated the tumor microenvironment by recruiting TAMs to glioblastoma tissues, leading to tumor growth (Fig. 7h). These findings reveal opportunities for research on the role of SETDB1 in disease progression.

SETDB1 functions as a histone methyltransferase to cause histone H3K9 trimethylation, which is involved in the formation of heterochromatin [38]. These H3K9 and H3K27 sites are connected to transcriptional regulation and epigenetics [39]. This presents an opportunity to target epigenetic modifiers such as SETDB1 to treat malignancies. Research has identified the overexpression of SETDB1 in many malignancies, such as glioblastoma, melanoma, prostate cancer, and breast cancer (BRC), which was linked to cancer cell division as well as metastasis [23, 26, 38]. Previously study have shown that SETDB1 in macrophages potently suppresses Toll-like receptor 4 (TLR4)-mediated expression of proinflammatory cytokines including interleukin-6 through its methyltransferase activity [40]. However, a complete picture is lacking in this area of cancer studies.

Our study focuses on the association of TAMs with cancer cells in the tumor microenvironment [41, 42]. These cells have been shown to synthesize several factors that modulate cancer cell division and angiogenesis according to recent studies [43]. Particularly, the presence of symbiosis between macrophages and tumor cells has been shown by experiments where coculture of these cells caused the degradation of collagen [44]. Previous study has shown that macrophage recruitment plays a key role in GABRP-mediated tumor progression in pancreatic cancer [45]. TAMs also involved in tumor growth in glioblastoma [45, 46]. The results from this work highlight several novel features of the mechanisms underlying glioblastoma. Such features of TAMs facilitate research targeting these cells in response to disease. CSF-1 and its receptor, colony-stimulating factor 1 receptor (CSF-1R), are areas of concern and are being developed in clinical research [47]. One feature that is encouraging here is identification of safe applications of immunotherapeutic or standard treatment tools [48–50]. Such promising activity has been demonstrated in autocrine CSF-1-based benign diffuse-type tenosynovial giant cell tumors [51, 52]. In the case of malignant disorders, reports from clinical perspectives have yet to be explored.

RETRACTED

Continuous research facilitates the understanding that distinct macrophage features, such as functions and phenotypes, are a reflection of various signals (for differentiation, polarization, survival or recruitment) in a tissue-specific environment [53]. The implication here is that targeting TAMs for therapy would show variation according to the organ in which the cells are present [54, 55]. This work showed that SETDB1 promotes CSF-1 induction and secretion by tumor cells and CSF-1 is involved in tumor progression and TAM infiltration. The origin of CSF-1 can be traced back to circulating monocytes in the blood vessels of the tumor. This provides the possibility that CSF-1 and its sustained production could serve as a target for efficient disease treatment. Consistence with previous study [56], our findings showed that the increase in SETDB1 promotes CSF-1 induction via AKT/mTOR activation. Interestingly, our results also demonstrated that silencing of AKT also reduces CSF-1 levels, in both U87 and U251 cell lines (Fig. 5c and d). Therefore, our findings indicated that AKT may induce CSF-1 expression independently of SETDB1. Hence, this work proposes a molecular mechanism for CSF-1 overexpression in glioblastoma, opening up the possibility for this molecule or its receptor to be a target in patients with SETDB1-overexpressing glioblastoma. In this study, we used two mouse model, xenograft and syngeneic mouse model, which were established from intrathecal cancer cell injection. Due to the cancer cells are injected in a place with a completely different tumor microenvironment, very far from tumor microenvironment can be found in the CNS. Therefore, orthotopic tumor model is needed to confirm our results in the future.

## Conclusion

In the current study, our findings indicated that SETDB1 upregulated in glioblastoma and relative to poor progression. Overexpression of SETDB1 promotes proliferation, invasion and migration. Our findings also indicated that SETDB1 promotes macrophage recruitment and polarization via AKT/mTOR-dependent CSF-1 induction and secretion. Our results indicated that SETDB1 is essential for glioblastoma tumorigenesis, and may be a newly target for treatment and prognostic evaluation in glioblastoma, which will be the focus of our future investigations.

RETRACTED

## Supplementary information

**Additional file 1.**

## Data Availability

All data generated or analyzed during this study are included in this published article.

## Abbreviations

ATCC: American Type Culture Collection
BSA: Bovine serum albumin
CM: Conditioned media
CNS: Central nervous system
CSF-1: Colony stimulating factor 1
CSF-1R: Colony-stimulating factor 1 receptor
DMEM: Dulbecco’s modified Eagle’s medium
ELISA: Enzyme-linked immunosorbent assay
EV: Empty vector
FBS: Fetal bovine serum
IHC: Immunohistochemistry
NHAs: Normal human astrocytes
OS: Overall survival
PVDF: Polyvinylidene fluoride
SD: Standard deviation
SETDB1: SET domain bifurcated 1
TAMs: Tumor-associated macrophages
TMZ: Temozolomide
